The article "Preoperative Predictors of Prolonged Hospital Stay in Accelerated Rehabilitation for Patients Undergoing Orthopedic Surgery" was retracted in 2023. Reasons: signs of a paper mill; suspected computer-generated content; unreliable results or conclusions; lack of ethics approval or compliance.

# Preoperative Predictors of Prolonged Hospital Stay in Accelerated Rehabilitation for Patients Undergoing Orthopedic Surgery

**DOI:** 10.1155/2021/7832216

**Published:** 2021-11-19

**Authors:** Shu Huang, Yong Xie, Zhiyan Huang, Jiangyi Wu, Junjun Yang, Qiaoyin Tan, Guanyu Chen, Jun Yuan, Xiaoni Liu, Hui Wu, Baorong Liu, Yizhao Zhou, Sihong Li, Xiaosheng Li, Guimin Zhang, Xiangyang Liu, Jing Wang

**Affiliations:** ^1^Department of Orthopedics, Hunan Provincial People's Hospital (The First-affiliated Hospital of Hunan Normal University), Changsha 410005, China; ^2^Lunan Pharmaceutical Group Co. Ltd., Linyi 276000, China; ^3^State Key Laboratory of Generic Manufacture Technology of Chinese Traditional Medicine, Linyi 276000, China; ^4^Peking University Shenzhen Hospital, Shenzhen 518000, China; ^5^Key Laboratory of Biorheological Science and Technology, Ministry of Education College of Bioengineering, Chongqing University, Chongqing 400044, China; ^6^College of Teacher Education, Zhejiang Normal University, Jinhua 321004, China

## Abstract

In this study, we performed a retrospective and prospective study of preoperative predictors of the length of stay (LOS) in three groups of surgical patients and conducted a clinical retrospective study of the current research status of preoperative predictors of LOS prolongation in three groups of patients under ERAS (enhanced recovery after surgery) mode, such as patient characteristics and comorbidities. Information such as patients' exercise preferences, exercise time, frequency and duration, footwear, location of knee osteoarthritis, whether there is a past history of knee injury, and smoking and drinking history was collected, and the research data of 312 patients undergoing the three operations were analyzed by SPSS. Meniscal injury-knee arthroscopy sample included a total of 104 people. Surgical sample for anterior cruciate ligament reconstruction included a total of 100 subjects. Knee osteoarthritis-knee replacement surgery sample included 148 people who were divided into two groups in a ratio of 1 : 1: one group used Mailuo Shutong pills during hospitalization (intervention group) and the other group did not (control group). The research conclusions are as follows. *Meniscal Knee Arthroscopy*. (1) Samples from different causes of injury showed significant differences for all injured sites. (2) Samples with different smoking and drinking histories all showed significant differences for the causes of injury. (3) Exercise hobby, exercise frequency, duration of each exercise and duration of exercise, and warm-up time before exercise all showed positive correlation. *Anterior Cruciate Ligament Reconstruction Surgery*. (4) Samples from different causes of injury showed significant differences for all the injured sites. (5) Age has a significant negative influence on the wearing of shoes at ordinary times. (6) Exercise hobby: the warm-up time before exercise had a significant negative influence on the injured area. (7) Two groups of analysis items of exercise frequency, exercise duration and exercise duration, preexercise warm-up time, and exercise hobby were typically positively correlated. *Total Knee Arthroplasty*. (8) There was a significant difference of 0.01 between the hospitalization days of the intervention group and the control group (*p* < 0.01), and the hospitalization days of the intervention group were significantly lower than those of the control group. These results indicated that Mailuo Shutong pills were of great significance for the treatment of orthopedic patients during the operation period in that it could effectively shorten the hospital stay of all orthopedic patients and strengthen the accelerated rehabilitation. (9) There was a significant positive correlation between the history of knee joint surgery and the use time of Mailuo Shutong pills. (10) There was a markable positive correlation between occupation and sports hobbies, sports time, frequency and duration, and footwear. There was a significant negative correlation between occupation and preexercise warm-up. (11) Exercise time, frequency, and duration have significant positive influence on BMI.

## 1. Introduction

The enhanced recovery after surgery (ERAS) model is an important tool in medical application [1,2]. Yazdchi et al. [3] performed a ERAS cardiac surgery for a propensity-matched analysis. Li et al. [4] used the ERAS model in prediction of risk for ovarian cancer patients. Lindenmuth et al. [5] used the ERAS model in implantation with ventricular assist device. These models show interesting and important findings which benefit the medical applications. With the extensive application of the ERAS model, the length of stay (LOS) of patients has also been studied [6].

The meniscal knee arthroscopy is a medical technique for doctors directly seeing through meniscus of knee joint via arthroscope [7,8]. Antunes et al. [9] studied the knee meniscal injuries for correlation with video arthroscopy. Ciccotti et al. [10] worked on the prevalence of articular cartilage changes using the technique. Anterior cruciate ligament reconstruction surgery is a minimally invasive surgery under arthroscope for the sports injury [11–13]. Saini et al. [14] compared the combined adductor canal block with perihamstring infiltration versus adductor canal block for postoperative analgesia in arthroscopic anterior cruciate ligament reconstruction surgery. Kaur et al. [15] studied the surgery effect after 2–10 years. Zhang et al. [16] studied the efficacy of an imaging system for the technique. The total knee arthroplasty is a new technique for treating knee joint diseases developed gradually after the successful application of artificial hip joint [17–19]. Zhong et al. [20] studied mirabilite after TKA. Alessi et al. [21] studied the functionality of a robotic surgical assistant for TKA. These techniques can be improved with current ERAS and other mathematical models and analysis.

In a general sense, LOS can be significantly shortened with ERAS model, in this work, for the meniscal knee arthroscopy, anterior cruciate ligament reconstruction surgery, and total knee arthroplasty (TKA). Mailuo Shutong pills (Wan in Chinese) [22,23] are of great significance for the perioperative treatment of orthopedic patients, which can effectively shorten the hospitalization time of orthopedic patients, strengthen and accelerate rehabilitation, prevent and treat DVT of lower limbs, and enhance the satisfaction rate of patients and their families. The main risk factors of knee osteoarthritis patients [24,25] may be (or related to) obesity, rural residents, age, previous history of trauma, heredity, smoking, female (menopause), etc. The risk factors of patients with anterior cruciate ligament (ACL) [26] exercise mainly include women (before menopause), urban residents, previous history of trauma, no warm-up, irregular exercise, etc. The main risk factors of patients with meniscus injury [27–29] are male, urban residents, previous history of trauma, lack of warm-up, weight, age (≤40 years old), etc. The mathematical tools are important methods in medical studies [30–32]. In this study, we performed a retrospective and prospective study of preoperative predictors of the length of stay (LOS) in three groups of surgical patients and conducted a clinical retrospective study of the current research status of preoperative predictors of LOS prolongation in three groups of patients under ERAS (enhanced recovery after surgery) mode, such as patient characteristics and comorbidities. Information such as exercise hobby, time, frequency and duration of exercise, footwear, location of knee arthritis, whether there was a past history of knee injury, and smoking and drinking history of the patients was collected and analyzed with SPSS.

## 2. Objective and Methods

Information such as patients' exercise preferences, exercise time, frequency and duration, footwear, location of knee osteoarthritis, whether there is a past history of knee injury, and smoking and drinking history was collected. The research data of 312 patients undergoing the three operations (meniscus knee arthroscopy, anterior cruciate ligament reconstruction, and total knee arthroplasty) were analyzed by SPSS.

Meniscal injury-knee arthroscopy sample included a total of 104 people.  Table 1 shows that the percentage of women is 55.77% for both sexes. The proportion of male samples was also 44.23%.

Surgical sample for anterior cruciate ligament reconstruction included a total of 100 subjects.  Table 2 shows that the total number in the sample is 100, and the proportion of choosing “male” is 81.00% and that of female is 19.00%.

Knee osteoarthritis-knee replacement surgery sample included 148 people who were divided into two groups in a ratio of 1 : 1: one group used Mailuo Shutong pills during hospitalization (intervention group) and the other group did not (control group).  Table 3 shows that in the intervention group, the sex/female ratio was 64.86%. The proportion of male samples was 35.14%. The percentage of females in the control group was 66.22%, and the proportion of male samples was 33.78%.

## 3. Results and Discussion

### 3.1. Meniscus Injury-Knee Arthroscopy

Meniscal injury: 104 samples were examined by arthroscopy.

Normality test for age was performed, and it can be seen from Table 4 that the sample sizes of study data were all greater than 50, so the KS test was used. Specifically, all ages showed no significant difference (*p* > 0.05), which meant that the original hypothesis (original hypothesis: normal distribution of data) was accepted, and all ages showed normal characteristics.

Table 5 exhibits the relationship between the causes of injury (sports trauma, other trauma, and no history of trauma) and the injured site: artificial grassland, grassland, artificial floor, wood floor, cement floor, and floor tile. From the above table, it can be seen that samples with different causes of injury showed significant differences for the injured site (*p* < 0.05). It is specifically recommended that the differences be compared in combination with the percentages in brackets. The cause of injury (sports trauma, other trauma, and no history of trauma) showed 0.01-level significance for the injured site: artificial grassland, grassland, artificial floor, wood floor, cement floor, and floor tile (chi = 69.254, *p* ≤ 0.01). According to the difference in percentage comparison, the proportion of patients with no obvious injury and those with no choice was 71.43%, which was significantly higher than the average level of 28.85%. 100% cases of playing basketball are injured on the cement floor, which is significantly higher than the average level 64.42%. (see Figure 1 for details).

*Summary*. Samples with different causes of injury (sports trauma, other trauma, and no history of trauma) showed significant differences for all of the injured sites: artificial grassland, grassland, artificial floor, wood floor, cement floor, and floor tile.

Table 6 displays the relationship between smoking and drinking history and the injury cause. From the above table, it can be seen that different smoking and drinking history samples showed significant effects on the injury cause (*p* < 0.05).

As can be seen from the percentage comparison difference, 55.56% of smokers who chose not to have obvious injury history will be obviously higher than the average level of 40.38%. The proportion of alcohol users who chose not to have obvious injury history was 50.00%, which was obviously higher than the average level of 40.38%. 63.64% of the patients, who sprain their knee, have habits of smoking and alcohol-drinking. The percentage was higher than the average level 42.31%. It was concluded that among the samples with different smoking and drinking histories, all causes of injury showed significant differences.

As shown in Table 7, Pearson correlation coefficient was used to study the correlation among exercise hobby, exercise frequency, duration of each exercise and duration of exercise, and warm-up time before exercise.

The correlation coefficient values were 0.412 and 0.472, respectively, and the correlation coefficient values were all greater than 0, suggesting that there was a positive correlation between exercise hobby and exercise duration and warm-up time before exercise. Significant correlations were found between exercise frequency, exercise duration, and preexercise warm-up time, with correlation coefficient values of 0.803 and 0.549, respectively. The coefficient value > 0 shows that the exercise frequency is positively correlated with exercise time and warm-up time before exercise. The correlation coefficient values of duration of each exercise were 0.764 and 0.529, respectively, for the groups of duration of exercise and pre-exercise warm-up time, and the correlation coefficient values were greater than 0, indicating that there was a positive correlation between duration of each exercise and duration of exercise and preexercise warm-up time.

### 3.2. Anterior Cruciate Ligament Injury-Anterior Cruciate Ligament Reconstruction Surgery

Surgical sample for anterior cruciate ligament reconstruction included a total of 100 subjects.

Table 8 displays the differential relationship between the cause of injury and the injured site. It shows the samples with different causes of injury had a significant effect on the injured field (*p* < 0.05) (chi = 488.238). By comparing the percentages, we could find that the proportion of playing football on artificial grassland was 91.67%, which was significantly higher than the average level of 11.00%. The percentage of playing table tennis with plastic flooring was 100.00%, which was significantly higher than the average level of 17.00%. The proportion of playing badminton with plastic floor is 50.00%, which is obviously higher than the average level of 17.00%. 100.00% of runners chose concrete floors, which was significantly higher than the average of 56.00%. The proportion of heavy objects striking the selected concrete floor was 100.00%, which would be significantly higher than the average level of 56.00%. In conclusion, samples with different causes of injury showed significant differences for all injured sites.

Table 9 shows that linear regression analysis was performed with age as independent variable and shoes as dependent variable. The model formula was as follows: shoes worn at ordinary times = 15.870–0.176∗ age, and the square value of model *R* was 0.092, indicating that age could explain 9.2% change of shoes worn at ordinary times. The model's *F*-test shows that the model passed (*F* = 9.982, *p*=0.002 < 0.05), which means that age definitely has an impact on the shoes you usually wear. The regression coefficient value of age was −0.176 (*t* = −3.159, *p*=0.002 < 0.01), which meant that age had a significant negative influence on the shoes worn.

Table 10 shows that exercise hobby, duration of each exercise, warm-up time before exercise, exercise frequency, and duration of exercise are taken as independent variables, and the injured site is taken as dependent variable for stepwise regression analysis. After the automatic recognition of the model, finally the remaining sports hobbies and the preexercise warm-up time were two items in total in the model. Model formula: injured site = 7.427–0.089∗ exercise hobby −0.087∗ warm-up time before exercise, and *R*-square value is 0.123, which means exercise hobby. The warm-up time before exercise can explain 12.3% change reason of injured site. Moreover, the model passed the *F*-test (*F* = 6.795, *p*=0.002 < 0.05), indicating that the model was effective. In addition, the multicollinearity of the model is tested, and it is found that all the VIF values in the model are less than 5, which means that there is no collinearity problem. The value of D-W is near the number 2, which indicates that the model has no autocorrelation and there is no correlation between the sample data, so the model is good. The final specific analysis shows that the regression coefficient value of exercise hobbies was −0.089 (*t* = −2.475, *p*=0.015 < 0.05), and the regression coefficient value of warm-up time before exercise was −0.087 (*t* = −2.284, *p*=0.025 < 0.05), which indicated that exercise hobbies and warm-up time before exercise had a significant negative impact on the injured site.

As shown in Table 11, the typical correlation analysis was used to study the typical correlation between the duration of each exercise, the warm-up time before exercise, the exercise hobby (three items) and the exercise frequency, and the duration of exercise (two items). As shown in the above table, two pairs of typical variables were extracted, which were analyzed specifically for the typical correlation coefficient. There were two typical correlation coefficient values in all and they were both significant (*p* < 0.05). The two typical correlation coefficient values were 0.667 and 0.373, respectively. A positive number indicated a positive correlation, indicating that there was a typical positive correlation between the two analysis items in this study: *X* (exercise frequency and exercise duration) and *Y* (exercise duration, preexercise warm-up time, and exercise hobby).

### 3.3. Knee Osteoarthritis-Knee Replacement

Knee osteoarthritis-knee replacement surgery sample included 148 people who were divided into two groups in a ratio of 1 : 1: one group used Mailuo Shutong pills during hospitalization (intervention group) and the other group did not (control group).

As shown in Table 12, the hospital stay of the two groups was paired, and Wilcoxon signed rank sum test was used to study the hospital stay, and the paired data showed differences (*p* < 0.05). There was a significant difference at the 0.01 level between the hospitalization days of the intervention group and the control group (*p* < 0.01), and the median hospitalization days of the intervention group (11.000) were significantly lower than those of the control group (17.000). Next, the experimental data of the intervention group were analyzed in detail.

As shown in Table 13, the Pearson correlation coefficient was used to represent the strength of the relationship between the intervention group's previous history of knee surgery and the use time of Mailuo Shutong pills. The correlation coefficient value was 0.252, and there was significant difference at 0.05 level. It is suggested that there is a markable positive correlation between the history of knee joint surgery and the use time of Mailuo Shutong pills.

Table 14 shows the Pearson correlation of occupation for “sports hobby,” “time, frequency, and duration of exercise,” “footwear,” and “is there a warm-up before exercise?” Pearson correlation coefficient was used to analyze the relationship between the variables. The coefficient value between occupation and sports hobby was 0.235, *p* < 0.05. The coefficient values between occupation and exercise time, frequency, and duration were 0.292 (*p* < 0.05). The coefficient between occupation and footwear was 0.272, *p* < 0.05. Therefore, it indicated that occupation had significant positive correlation with exercise hobby, exercise time, frequency and duration, and footwear. The correlation coefficient between occupation and whether to warm up before exercise was −0.403, *p* < 0.01. Therefore, there is a significant negative correlation between occupation and whether there is warm-up before exercise.

Table 15 shows the time, frequency, and duration of exercise as independent variables and BMI as dependent variable. The model formula was as follows: BMI = 23.821 + 0.193∗ exercise time, frequency, and duration of years. The R-square of the model was 0.079, and exercise time, frequency, and duration of years could explain the 7.9% change in BMI. The *F*-test of the model showed that the model passed the *F*-test (*F* = 6.203, *p*=0.015 < 0.05), which meant that the exercise time, frequency, and duration of years must have an impact on BMI.

Through in-depth analysis, we could find that the regression coefficient values of exercise time, frequency, and duration of years were 0.193 (*t* = 2.491, *p*=0.015 < 0.05), which meant that exercise time, frequency, and duration of years had a significant positive impact on BMI.

## 4. Conclusions

*Meniscal Knee Arthroscopy*. (1) Samples from different causes of injury showed significant differences for all injured sites. (2) Samples with different smoking and drinking histories all showed significant differences for the causes of injury. (3) Exercise hobby, exercise frequency, duration of each exercise and duration of exercise, and warm-up time before exercise all showed positive correlation.

*Anterior Cruciate Ligament Reconstruction Surgery*. (4) Samples from different causes of injury showed significant differences for all the injured sites. (5) Age has a significant negative influence on the wearing of shoes at ordinary times. (6) Exercise hobby: the warm-up time before exercise had a significant negative influence on the injured area. (7) Two groups of analysis items of exercise frequency, exercise duration and exercise duration, preexercise warm-up time, and exercise hobby were typically positively correlated.

*Total Knee Arthroplasty*. (8) There was a significant difference of 0.01 between the hospitalization days of the intervention group and the control group (*p* < 0.01), and the hospitalization days of the intervention group were significantly lower than those of the control group. These results indicated that Mailuo Shutong pills were of great significance for the treatment of orthopedic patients during the operation period in that it could effectively shorten the hospital stay of all orthopedic patients and strengthen the accelerated rehabilitation. (9) There was a significant positive correlation between the history of knee joint surgery and the use time of Mailuo Shutong pills. (10) There was a significant positive correlation between occupation and sports hobbies, sports time, frequency and duration, and footwear. There was a significant negative correlation between occupation and preexercise warming-up. (11) Exercise time, frequency, and duration have significant positive influence on BMI.

## Figures and Tables

**Figure 1:** Injury etiology and injury site.

**Table 1:** Basic analysis (*n* = 104).

Project	Option	Frequency	Percentage	Cumulative percentage
Gender	Female	58	55.77	55.77
	Male	46	44.23	44.23

Sum		104	100.0	100.0

**Table 2:** Frequency analysis.

Name	Option	Frequency	Percentage	Cumulative percentage
Gender	Female	19	19.00	19.00
	Male	81	81.00	81.00

Sum		100	100.0	100.0

**Table 3:** Frequency analysis.

Name	Option	Frequency	Percentage	Cumulative percentage
Intervention group gender	Female	48	64.86	64.86
	Male	26	35.14	35.14

Control group gender	Female	49	66.22	66.22
	Male	25	33.78	33.78

Sum		74	100.0	100.0

**Table 4:** Normality test analysis.

Name	Sample size	Average value	Standard deviation	Skewness	Kurtosis	Kolmogorov–Smirnov	Shapiro–Wilk	*W* value	*p*
						*D* value	*p*		
Age	104	21.212	10.952	0.037	−0.991	0.074	0.168	0.971	0.021^∗^

^*∗*^ *p* < 0.05.

**Table 5:** Cross-over (chi-square) analysis.

Subject	Name	Etiology of injury (motor trauma, other trauma, no history of trauma)							Percentage	*χ*²	*p*
		Play basketball	Fall	Crush injury	No obvious injury history	Sprain of knee	Run	Hurt by riding a bike			
Injured site	Plastic floor	0	0	0	0	6.82%	0	0	2.88	69.254	≤0.001^*∗∗*^
	Hilly area	0	0	0	0	4.55%	0	0	1.92		
	None	0	0	0	71.43%	0	0	0	28.85		
	Cement	100%	90.91%	100%	28.57%	86.36%	100%	100%	64.42		
	Earth floor	0	9.09%	0	0	2.27%	0	0	1.92		
	Number of cases	3	11	2	42	44	1	1	104		

^*∗∗*^ *p* < 0.01.

**Table 6:** Cross-over (chi-square) analysis.

Subject	Name	History of smoking and drinking				Amount to	*χ* ^2^	*p*
		Drink	Smoke	Smoking and drinking	Without			
Injury etiology	Playing basketball	0.00%	0.00%	0.00%	3.66%	2.88%	45.854	≤0.001^∗∗^
	Fall	0.00%	11.11%	0.00%	12.20%	10.58%		
	Crush injury	50.00%	0.00%	9.09%	0.00%	1.92%		
	No obvious injury history	50.00%	55.56%	27.27%	40.24%	40.38%		
	Sprain of knee	0.00%	22.22%	63.64%	42.68%	42.31%		
	Run	0.00%	11.11%	0.00%	0.00%	0.96%		
	Hurt by riding a bike	0.00%	0.00%	0.00%	1.22%	0.96%

Number of cases		2	9	11	82	104

^*∗∗*^ *p* < 0.01.

**Table 7:** Pearson correlations.

	Sports hobbies (running, football, basketball, etc.)	Exercise frequency (several times per week)	Duration of each exercise (hours)
Duration of exercise (years)	0.412^∗^	0.803^∗^	0.764^∗^
Warm-up time before exercise (minutes)	0.472^∗^	0.549^∗^	0.529^∗^

^∗^indicates high correlation.

**Table 8:** Cross-over (chi-square) analysis.

Subject	Name	Injury etiology													Amount to	*χ* ^2^	*p*
		Playing table tennis	Playing volleyball	Playing basketball	Playing badminton	Fall	None	Ski	Taekwondo	Run	Dance aerobics	Playing football	Traffic accident	Heavy impact			
Injured site	Artificial grassland	0	0	0	0	0	0	0	0	0	0	11	0	0	11	488.238	≤0.001^∗∗^
	Plastic floor	1	1	10	4	1	0	0	0	0	0	0	0	0	17		
	Without	0	0	0	0	0	2	0	0	0	0	0	0	0	2		
	Floorboard	0	0	4	1	0	0	0	0	0	0	0	0	0	5		
	Wooden floor	0	0	1	0	0	0	0	0	0	1	0	0	0	2		
	Unknown	0	0	0	0	0	1	0	0	0	0	0	0	0	1		
	Asphalt pavement	0	0	0	0	2	0	0	0	0	0	0	1	0	3		
	Cement floor	0	3	21	3	24	0	0	0	2	0	0	2	1	56		
	Foam pad	0	0	0	0	0	0	0	1	0	0	0	0	0	1		
	Lawn	0	0	0	0	0	0	0	0	0	0	1	0	0	1		
	Snow field	0	0	0	0	0	0	1	0	0	0	0	0	0	1		

Number of cases		1	4	36	8	27	3	1	1	2	1	12	3	1	100

^*∗∗*^ *p* < 0.01.

**Table 9:** Linear regression analysis (*n* = 100).

	Nonstandardized coefficient	Normalization coefficient		*t*	*p*	VIF	*R*²	Adjust *r*	*F*
	*B*	Standard error	Beta						
Constant	15.870	1.008	–	15.738	≤0.001^*∗∗*^	–	0.092	0.083	*F* (1,98) = 9.982, *p*=0.002
Age	−0.176	0.056	−0.304	−3.159	0.002^*∗∗*^	1.000			

Dependent variable: shoe type normally worn; D-W value: 1.949; ^*∗∗*^*p* < 0.01.

**Table 10:** Stepwise regression analysis (*n* = 100).

	Nonstandardized coefficient	Normalization coefficient		*t*	*p*	VIF	*R*²	Adjust *r*	*F*
	*B*	Standard error	Beta						
Constant	7.427	0.541	—	13.730	≤0.001^*∗∗*^		0.123	0.105	*F *(2,97) = 6.795, *p*=0.002
Sports hobby	−0.089	0.036	−0.239	−2.475	0.015^*∗*^	1.028			
Warm-up time before exercise (minutes)	−0.087	0.038	−0.220	−2.284	0.025^*∗*^	1.028			

Dependent variable: injured site; D-W value: 1.763; ^*∗∗*^*p* < 0.05; ^*∗∗*^*p* < 0.01.

**Table 11:** Typical correlation coefficient and significance.

Typical correlation pair	Canonical correlation coefficient	Wilks' lambda	*df 1*	*df 2*	*F*	*p*
1	0.667	0.478	6.000	190.000	14.139	≤0.001^∗∗^
2	0.373	0.861	2.000	96.000	7.750	≤0.001^∗∗^

^*∗∗*^ *p* < 0.01.

**Table 12:** Wilcoxon analysis results for paired samples.

name	Paired (median)		Difference (pair 1-pair 2)	Statistical value z	*p*
	Pair 1	Pair 2			
Days of hospitalization in the intervention group paired with those in the control group	11.000	17.000	−6.000	5.684	≤0.001^∗∗^

^*∗∗*^ *p* < 0.01.

**Table 13:** Pearson correlations.

		Any previous history of knee surgery
Usage time of Mailuo Shutong pills	Correlation coefficient	0.252^∗^
	*p* value	0.030

^*∗*^ *p* < 0.05.

**Table 14:** Pearson correlation.

	Occupation
Sports hobby	0.235^∗^
Time, frequency, and duration of exercise	0.292^∗^
Is there a warm-up before exercise	−0.403^∗∗^
Footwear	0.272^∗^

^*∗*^ *p* < 0.05; ^*∗∗*^*p* < 0.01.

**Table 15:** Linear regression analysis (*n* = 74).

	Nonstandardized coefficient	Normalization coefficient		*t*	*p*	VIF	*R*²	Adjust *r*	*F*
	*B*	Standard error	Beta						
Constant	23.821	0.476	—	49.999	≤0.001^*∗∗*^	—	0.079	0.067	*F *(1,72) = 6.203, *p*=0.015
Time, frequency, and duration of exercise	0.193	0.078	0.282	2.491	0.015^*∗*^	1.000			

Dependent variable: BMI; D-W value: 1.630; ^*∗*^*p* < 0.05; ^*∗∗*^*p* < 0.01.

## Data Availability

The data supporting this work are included within the article and the supplementary files.

## Supplementary Materials

Supplementary Materials (1) Raw data for anterior cruciate ligament injury-anterior cruciate ligament reconstruction surgery. (2) Raw data for the knee osteoarthritis-knee replacement in intervention group and control group. (3) Raw data for meniscus injury-knee arthroscopy.
